The article "Inhibiting Autophagy Pathway of PI3K/AKT/mTOR Promotes Apoptosis in SK-N-SH Cell Model of Alzheimer's Disease" was retracted in 2023. Reason: concerns about the peer review.

# Inhibiting Autophagy Pathway of PI3K/AKT/mTOR Promotes Apoptosis in SK-N-SH Cell Model of Alzheimer's Disease

**DOI:** 10.1155/2022/6069682

**Published:** 2022-02-08

**Authors:** Yu Pang, Wennan Lin, Lan Zhan, Jiawen Zhang, Shicun Zhang, Hongwei Jin, He Zhang, Xiaoli Wang, Xiaoming Li

**Affiliations:** ^1^Department of Neurology, The Second Affiliated Hospital of Qiqihar Medical University, Qiqihar 161000, China; ^2^General Department, The Second Affiliated Hospital of Qiqihar Medical University, Qiqihar 161000, China; ^3^School of Pharmacy, Qiqihar Medical University, Qiqihar 161000, China; ^4^The Institute of Medicine, Qiqihar Medical University, Qiqihar 161000, China

## Abstract

Alzheimer's disease is the most common dementia disease characterized by chronic progressive neurodegeneration. The incidence of Alzheimer's disease is on the rise as the population ages at an accelerating pace. According to epidemiological data, by 2050, the number of Alzheimer's patients in the United States will be three times higher than that in 2010, and a similar trend is occurring in China. To explore the effect and mechanism of let-7b by detecting the expression level of let-7b in Alzheimer's disease, fifty patients with Alzheimer's disease and thirty healthy controls were selected. The expression levels of let-7 families (let-7a, let-7b, let-7c, let-7d, let-7e, let-7f, let-7g, and let-7i) were detected by qPCR. Human neuroblastoma cell SK-N-SH were divided into control group (untreated), model group (treated with A*β*1-40), A*β*1-40+let-7b mimic group (treated with A*β*1-40 and transfected with let-7b mimic), and A*β*1-40+miR-NC group (treated with a*β*1-40 and transfected with miR-NC). let-7b expression and cell survival rate were detected by qPCR and CCK-8, and the levels of caspase 3, LC3, beclin-1, PI3K, p-AKT, and p-mTOR were detected by Western blot. let-7b was significantly different between the case group and the control group (*p* < 0.001). CCK-8 showed a significant decrease in cell viability in A*β*1-40 treatment group compared with that in the control group (*p* < 0.01). Overexpression of let-7b significantly reduced the survival rate of the cells, and the expression of LC3II/LC3I and beclin-1 in the cells was significantly reduced by a*β*1-40 treatment (*p* < 0.001). let-7b overexpression also inhibited autophagy via reducing the level of LC3II/LC3I and beclin-1 (*p* < 0.001). A*β*1-40 treatment and let-7b overexpression promoted apoptosis by increasing the expression of cleavage caspase 3. Western blot indicated that A*β*1-40 treatment and let-7b overexpression could increase the expression of PI3K, p-AKT, and p-mTOR. let-7b overexpression could inhibit autophagy and promote apoptosis in Alzheimer's cells by promoting PI3K/AKT/mTOR signaling pathway. PI3K/AKT/mTOR signaling pathway is involved in the imbalance between autophagy and apoptosis.

The article "Inhibiting Autophagy Pathway of PI3K/AKT/mTOR Promotes Apoptosis in SK-N-SH Cell Model of Alzheimer's Disease" was retracted in 2023. Reason: concerns about the peer review.

## 1. Introduction

Alzheimer's disease is the most common dementia disease characterized by chronic progressive neurodegeneration [1]. The incidence of Alzheimer's disease is on the rise as the population ages at an accelerating pace. According to epidemiological data, by 2050, the number of Alzheimer's patients in the United States will be three times higher than that in 2010 [2], and a similar trend is occurring in China [3]. Alzheimer's disease is a leading cause of disability and death, which brings a heavy burden to society and families [4]. The main pathological changes are neurofibrillary tangles, senile plaque deposition, and nerve cell death [5]. The key component of senile plaque has been proved to be *β*-amyloid (A*β*) [6, 7]. Deposition of A*β*1-40 is a key event in the development of pathogenic A*β* from diffusion to core plaque maturation and is the basis for the development of neurotoxic plaques in AD [8].

In recent years, the role of autophagy in Alzheimer's disease has attracted a wide range of attention. Like other cells, neurons also accumulate toxic substances or damaged organelles such as mitochondria during senescence, which need to be cleared by autophagy to maintain proper intracellular homeostasis [9]. A recent study found that the expression of autophagy-related genes ATG1, ATG8a, and ATG18 in *Drosophila melanogaster* was downregulated with aging, and its subsequent neuronal dysfunction and Alzheimer's disease phenotype were considered to be related to the decrease of autophagy activity and overproduction of A*β*. There is considerable evidence that autophagy deficiency occurs in both animal models of Alzheimer's disease and patients with Alzheimer's disease. Autophagy is a risk factor for Alzheimer's disease [6]. Recent studies have shown that the defect of autophagy-lysosome pathway is a vital system for removing misfolded proteins or damaged organelles, so the reduction of autophagy contributes to the formation of A*β* plaques or neurofibrillary tangles [10]. Autophagy has several stages, including phagocytic cell membrane separation, phagocytic cell elongation, and random cytoplasmic content engulfment, as well as autophagy maturation and fusion with lysosomes [11]. Among all the regulatory factors of autophagy, mammalian target of rapamycin (mTOR) has been considered to play a key role in autophagy. When activated, mTOR negatively controls autophagy origin by blocking the UNC-51-like kinase (ULK)1/2 complex. ULK1/2 can be used as an autophagy inducer to regulate the Beclin1-VPS34 complex [12]. Autophagosomes can be formed from the activation of microtubule-associated protein 1 light chain 3*β* (LC3B) by phosphatidylethanolamine [13]. In addition, activated mTOR can phosphorylate UV radiation resistance-related gene proteins to inhibit autophagosome maturation [14]. Therefore, activated mTOR can inhibit the stage required for autophagosome biosynthesis.

The article "Inhibiting Autophagy Pathway of PI3K/AKT/mTOR Promotes Apoptosis in SK-N-SH Cell Model of Alzheimer's Disease" was retracted in 2023. Reason: concerns about the peer review.

MicroRNA (miRNA) are posttranscriptional regulatory non-protein coding RNAs that can affect physiological processes such as development, proliferation, inflammation, and apoptosis [15, 16]. According to epigenetic studies, miRNA is associated with age and cognitive changes [17, 18], and its abnormal expression is closely related to the pathogenesis of Alzheimer's disease. The let-7 miRNA family was first identified in *Caenorhabditis elegans*, which exists in multiple species 7. Known as classical developmental regulators, they participate in the regulation of various physiological and pathological events, such as cell proliferation, differentiation, apoptosis, immune response, tumorigenesis, and metastasis [19]. Dubinsky et al. reported that let-7 miRNA can promote autophagy of primary cortical neurons [20]. Besides, the expression of let-7b and let-7e was reported to be upregulated in cerebrospinal fluid (CSF) of Alzheimer's patients [21]. However, some scholars found that let-7d and let-7g were downregulated in plasma samples of Alzheimer's patients [22]. Till now, the effect of let-7 on autophagy in Alzheimer's disease has not been determined.

Based on the current research of autophagy and let-7 miRNA in Alzheimer's disease, human neuroblastoma SK-N-SH cell line treated with A*β*1-40 was used in this study to establish an *in vitro* model of Alzheimer's disease. This study aimed to investigate the role and the molecular mechanism of let-7b in Alzheimer's disease. In a word, this study suggests that A*β*1-40 can induce apoptosis of SK-N-SH cells. In addition, let-7b overexpression can increase the apoptosis of A*β*1-40 treated cells by damaging autophagy, in which process the PI3K/AKT/mTOR signaling pathway is involved. let-7b can be used as a promising target and tool for Alzheimer's disease treatment research, but the specific interaction target needs to be further studied. In addition, more samples are needed to ensure the reliability of the experimental results.

## 2. Materials and Methods

### 2.1. Materials

#### 2.1.1. Cases

CSF was collected from 50 patients with confirmed Alzheimer's disease, including 28 males and 22 females. Meanwhile, 30 healthy subjects of the same age were enrolled, including 16 males and 14 females. The informed consent of all subjects was obtained. Inclusion criteria were as follows: all patients (1) were diagnosed with Alzheimer's disease according to the Chinese Classification and Diagnostic Criteria for Mental Disorders (Third Edition), (2) are aged 55–80 years, and (3) were informed and gave consent for participation. Exclusion criteria were as follows: (1) patients with vascular dementia or dementia due to other causes, (2) patients with mental and consciousness disorders such as anxiety and depression or with other types of mental disorders, (3) elderly patients with benign amnesia, (4) patients with severe cardiovascular diseases and organic visceral lesions, and (5) patients who were unable to cooperate with the study.

The article "Inhibiting Autophagy Pathway of PI3K/AKT/mTOR Promotes Apoptosis in SK-N-SH Cell Model of Alzheimer's Disease" was retracted in 2023. Reason: concerns about the peer review.

#### 2.1.2. Cell Line Source

SK-N-SH cells are human neuroblastoma cells, which were purchased from the cell bank of the Chinese Academy of Sciences and preserved in our laboratory.

#### 2.1.3. Reagents

miRVana™ Paris kit and TaqMan MicroRNA reverse transcription kit were purchased from Thermo Fisher Scientific, China. Dulbecco's modified eagle's medium (DMEM), pancreatin, and fetal bovine serum (FBS) were purchased from Gibco. A*β*1-40 was purchased from GL Biochem (Shanghai) Ltd. let-7b mimic and random negative control miRNA (miR-NC) were purchased from Shanghai GenePharma Co., Ltd., with the following sequence: let-7b mimic, 5′-AAC CAC ACA ACC TAC TAC CTCA-3′; miR-NC 5′-UUC UCC CGU GAA GUC ACG UTT-3′. Insulin-like growth factor 1 (IGF-1) was purchased from Bachem AG, Switzerland. LY294002, a PI3K inhibitor, was purchased from Apexbio, USA; cell-counting kit-8 (CCK-8) was purchased from Tongren Chemical Industry, Japan. RIPA lysate was purchased from Beyotime Biotechnology Co., Ltd., Shanghai, China. A potable qPCR instrument was purchased from Equal, USA. ImageQuant LAS4000mini ultrasensitive chemiluminescence imager was purchased from GE company, USA. First antibodies PI3K, caspase 3, p-AKT, AKT, p-mTOR (S2448), mTOR, LC3, beclin-1, and *β*-actin were purchased from American Cell Signaling Technology Inc., with the Cat. nos. of #4255, #9662, #4060, #4685, and #5536, respectively. Goat anti-mouse and goat anti-rabbit secondary antibodies were purchased from Thermo Fisher Scientific.

### 2.2. Methods

#### 2.2.1. CSF Collection and Treatment

Lumbar puncture was performed on subjects in a sitting position, and 12 mL CSF was collected in a polypropylene tube, which was then shaken and centrifuged immediately after collection (1,600 g, room temperature, 10 minutes). Then, it was equally divided into 200 *μ*L and frozen at −80°C within 30 minutes after a lumbar puncture to avoid refreezing after thawing.

The article "Inhibiting Autophagy Pathway of PI3K/AKT/mTOR Promotes Apoptosis in SK-N-SH Cell Model of Alzheimer's Disease" was retracted in 2023. Reason: concerns about the peer review.

Total RNA was isolated according to the procedure of miRVana Paris RNA isolation kit. Thereafter, the CSF was diluted with an equal volume of 2x denatured solution. An equal volume of acid phenol : chloroform was added. After centrifugation for 10 minutes (15000 g), the aqueous layer was mixed with 1.25 times the volume of absolute ethyl alcohol. The samples were then washed in a filter cartridge and eluted in RNase-free water. RNA was quantified by nanophotometry.

miRNA was isolated from the total RNA following the protocol of the TaqMan MicroRNA reverse transcription kit. The level of miRNA was detected by qPCR, and the reaction conditions of qPCR were 95°C for 10 s in the first stage, followed by 40 cycles of 95°C for 5 s and 60°C for 30 s. The relative expression levels of related mRNA were calculated by 2^−△△CT^. See Table 1 for details.

#### 2.2.2. Cell Culture and Treatment

SK-N-SH cells were cultured in DEME containing 10% FBS, and the incubator conditions were controlled at a constant temperature of 37°C, 5% CO2, and saturated humidity. The culture medium was changed 1–2 times a week, and when the cells reached 90% confluence, they were digested and passaged with pancreatin. A*β*1-40 was dissolved in sterile PBS to prepare a solution with a concentration of 1 M. The solution was incubated at 37°C for 5 days to induce aggregation. Then, SK-N-SH cells with 4 × 10^5^ cells/well were inoculated in 6-well plates and then treated with A*β* 1–40 with a final concentration of 500 nm at 37°C for 7 days to establish an Alzheimer's disease model [23].

For different interventions, SK-N-SH cells were subdivided into four groups: normal control group, A*β*1-40 (model group: normal cells treated with A*β*1-40), A*β*1-40+let-7b mimic group (SK-N-SH cells treated with A*β*1-40 were transfected with 100 pM let-7b mimic), and A*β*1-40+miR-NC group (SK-N-SH cells treated with A*β*1-40 were transfected with 100 pM miR-NC).

#### 2.2.3. Determination of Cell Viability

Cell viability was determined by CCK-8 kit. After adding CCK-8 solution (10% of the culture medium volume) to each well of each group in the 96-well plates, the cells were incubated for 3 hours. Then, the absorbance value of each group of cells was measured at 450 nm, and the standard curve was obtained according to the standard. Then, the absorbance value of other groups was brought into the formula and converted to survival rate. The survival rate of the normal control group was set as 100%, and the relative survival rate of other groups was calculated.

#### 2.2.4. Western Blot

RIPA lysate was used to lyse cells, and a BCA kit was utilized to determine protein concentration. The sample loading amount was 30 ug, the separation gel concentration was 10%, and the gel running voltage was 80 V to 120 V in this experiment. A polyvinylidene fluoride (PVDF) membrane was applied, and the membrane was rotated at a constant pressure of 120 V, with mTOR for 3 hours and other proteins for 1 hour and 10 minutes. Then, the following first antibodies PI3K (1 : 1000), p-AKT (1 : 2000), AKT (1 : 1000), p-mTOR (1 : 1000), mTOR (1 : 1000), LC3 (1 : 1000), beclin-1(1 : 1000), caspase 3 (1 : 1000), and *β*-actin (1 : 1000) were added for incubation at 4°C overnight. After washing the membrane, the corresponding goat anti-mouse and goat anti-rabbit secondary antibodies (1 : 4000) were incubated, respectively, and then exposed and developed. Quantity One software was applied to analyze the gray value of the bands.

The article "Inhibiting Autophagy Pathway of PI3K/AKT/mTOR Promotes Apoptosis in SK-N-SH Cell Model of Alzheimer's Disease" was retracted in 2023. Reason: concerns about the peer review.

### 2.3. Statistical Analyses

The experimental results were all expressed as mean ± standard error (X ± SEM) and were statistically analyzed and plotted by Prism 7 software. qPCR results were analyzed by *t*-test, the other results were analyzed by one-way ANOVA, and the comparison between groups was performed by Bonferroni test. *p* < 0.05 (^*∗*^), *p* < 0.011 (^*∗∗*^), and *p* < 0.001 (^*∗∗∗*^) were considered to be statistically significant.

## 3. Results

### 3.1. Detection of microRNA in CSF of Patients with Alzheimer's Disease

Total RNA was extracted from CSF of controls and patients with Alzheimer's disease, and the expression of 8 microRNAs was detected. The results showed that compared with the control group, the expression of let-7b microRNA in the case group was significantly increased, with statistical significance (Figure 1).

The expression of 8 microRNAs was detected in cerebrospinal fluid of normal subjects of the same age and Alzheimer's patients, among which the expression of let-7b microRNA was found to be significantly increased.  ^*∗*^ ^*∗*^ ^*∗*^*p* < 0.001 versus control group.

### 3.2. Expression of let-7b in SK-N-SH Cells and Its Influence on Cell Viability

As shown in Figure 2(a), in SK-N-SH cells, the level of let-7b in A*β*1-40+ let-7b mimic group was significantly higher than that in A*β*1-40 group (*p* < 0.001).  Figure 2(b) demonstrated that A*β*1-40 treatment resulted in a significant reduction in cell viability compared with the control group (*p* < 0.01). In addition, let-7b overexpression significantly reduced SK-N-SH cell viability compared with A*β*1-40 group (*p* < 0.01).

### 3.3. Effect of let-7b on Autophagy and Apoptosis of SK-N-SH Cells Treated with A*β*1-40

The effect of let-7b on autophagy of SK-N-SH cells treated with A*β*1-40 was determined by detecting the expression levels of LC3II/LC3I and beclin-1. As shown in Figures 3(a)–3(b) compared with the control group, A*β*1-40 treatment resulted in significantly decreased LC3II/LC3I and beclin-1 levels in cells compared with the control group (*p* < 0.001). Compared with A*β*1-40 group, let-7b overexpression significantly reduced the expression levels of LC3II/LC3I and beclin-1 (*p* < 0.001), indicating that A*β*1-40 could inhibit autophagy, while let-7b overexpression could make autophagy inhibition worse. The effect of let-7b on apoptosis of SK-N-SH cells treated with A*β*1-40 was determined by analyzing the expression of cleavage caspase 3. As shown in Figures 3(a) and 3(d)), cleavage caspase 3 expression in cells treated with A*β*1-40 significantly increased compared with the control group (*p* < 0.001). Compared with A*β*1-40 group, let-7b overexpression significantly increased the expression level of cleavage caspase 3 (*p* < 0.001), indicating that A*β*1-40 can induce apoptosis, while overexpression of let-7b further enhanced the apoptosis. In addition, as shown in Figures 3(a), 3(e), 3(f), and 3(g)), the expression levels of PI3K, p-AKT, and p-mTOR in the upstream molecular pathway of autophagy were upregulated by A*β*1-40 and further elevated by let-7b overexpression, indicating that let-7b might inhibit autophagy by promoting PI3K/AKT/mTOR pathway, resulting in increased apoptosis in A*β*1-40 treated cells.

The article "Inhibiting Autophagy Pathway of PI3K/AKT/mTOR Promotes Apoptosis in SK-N-SH Cell Model of Alzheimer's Disease" was retracted in 2023. Reason: concerns about the peer review.

### 3.4. Effect of let-7b Inhibitor on PI3K/AKT/mTOR Signaling Pathway

To determine whether let-7b acts as a proapoptotic agent through the PI3K/AKT/mTOR pathway, we added LY294002, an inhibitor of let-7b, to test the changes of the above indexes [A*β*1-40+let-7b mimic + LY294002 group (cells were treated at 37°C with a final concentration of 25 *µ*M LY294002 for 48 hours)]. Compared with A*β*1-40+let-7b mimic group, LC3II/LC3I and beclin-1 in A*β*1-40+let-7b mimic + LY294002 group were upregulated (Figures 4(a)–4(c)), cleavage caspase 3 was downregulated (Figures 4(a) and 4(d)), and PI3K, p-AKT, and p-mTOR decreased (Figures 4(a), 4(e), 4(f), and 4(g)). The above results showed that LY29400, an inhibitor of let-7b, could significantly improve the increase of apoptosis and the decrease of autophagy induced by let-7b overexpression, and PI3K/AKT/mTOR signaling pathway was involved.

### 3.5. Effect of let-7b Agonist on PI3K/AKT/mTOR Signaling Pathway

In order to further determine whether let-7b plays a proapoptotic role through the PI3K/AKT/mTOR pathway, we added IGF-1, an agonist of let-7b, and then detected the changes of the above indexes (A*β*1-40+let-7b mimic + IGF-1 group (cells were treated at 37°C with a final concentration of 100 ng/ml IGF-1 for 48 hours)). It was found that LC3II/LC3 I and beclin-1 were downregulated (Figure 5(a)–5(c)), cleavage caspase 3 was upregulated (Figures 5(a) and 5(d)), and PI3K, p-AKT, and p-mTOR were upregulated (Figures 5(a), 5(e), 5(f), and 5(g)) in A*β*1-40+let-7b mimic + IGF-1 group as compared to A*β*1-40+let-7b mimic group. The above results demonstrated that IGF-1, an agonist of let-7b, could significantly aggravate the increase of apoptosis and the decrease of autophagy level caused by let-7b overexpression, and the PI3K/AKT/mTOR signaling pathway was involved.

The article "Inhibiting Autophagy Pathway of PI3K/AKT/mTOR Promotes Apoptosis in SK-N-SH Cell Model of Alzheimer's Disease" was retracted in 2023. Reason: concerns about the peer review.

## 4. Discussion

SK-N-SH cells induced by A*β*1-40 have been used as a neurotoxic model in a large number of previous studies [24, 25]. In this study, the cells were used as an *in vitro* model of Alzheimer's disease. It was confirmed that overexpression of let-7b promoted A*β*1-40 to induce the PI3K/AKT/mTOR pathway in SK-N-SH cells to inhibit autophagy and promote apoptosis.

There is increasing evidence that abnormal accumulation of A*β* may induce significant cytotoxicity in neurons and is the key pathogenic factor of Alzheimer's disease [26]. In this study, A*β*1-40 was used to investigate the mechanism of A*β* neurotoxicity. The main causes of Alzheimer's disease are A*β* tangles; therefore, treating SK-N-SH cells with A*β*1-40 can represent the cell model of Alzheimer's disease. The experimental results showed that cells treated with A*β*1-40 showed a significant decrease in cell viability and a significant increase in apoptosis rate compared to the control group, which was consistent with previous studies [24, 25]. In addition, let-7b overexpression further reduced the cell viability and enhanced the apoptosis level compared with A*β*1-40. These results indicated that overexpression of let-7b enhanced neurotoxicity induced by A*β*1-40 *in vitro*.

A recent study found that the expression of autophagy-related genes ATG1, ATG8a, and ATG18 in *Drosophila melanogaster* was downregulated with aging, and its subsequent neuronal dysfunction and Alzheimer's disease phenotype were considered to be related to the decrease of autophagy activity and overproduction of A*β* [27]. This suggests that age-induced reduction in autophagy-related gene expression is associated with late onset of Alzheimer's disease. Apolipoprotein E4 (ApoE4) is a major genetic risk factor for hereditary Alzheimer's disease, which can induce autophagy dysfunction. Overexpression of ApoE4 increased the amount of A*β*1-42 in mouse lysosomes and eventually led to the death of hippocampal neurons [28]. All these results indicate that overactivation of mTOR can lead to accumulation of A*β*. mTOR kinase pathway is a key regulator of autophagy, which is controlled by upstream PI3K/AKT pathway [28], and has a negative feedback effect on autophagy. Hence, inhibition of PI3K/AKT/mTOR pathway can activate autophagy [28]. Moreover, it can enhance lysosomal leakage and apoptosis caused by A*β* peptides in neuro-2a cells [29]. In addition, activated mTOR can phosphorylate UV radiation resistance-related gene proteins to inhibit autophagosome maturation [14]. Therefore, activated mTOR can inhibit the stage required for autophagosome biosynthesis. All of these indicate that autophagy is essential in Alzheimer's disease. Autophagy is regulated by various signal transduction pathways. Of these, mTOR, as a major negative regulator, is a protein kinase that senses the availability of cell energy and regulates cell proliferation. Reports show that mTOR signal is overactive in the brain regions of patients with Alzheimer's disease [30, 31]. Besides, it is shown that genetic reduction of mTOR in brain of Tg2576 mice results in the decrease of A*β* deposition and could save memory defects by increasing autophagy induction and restoring gene expression characteristics in the hippocampus [32]. In this study, the role of this pathway in autophagy was confirmed. Compared with controls, A*β*1-40 treatment upregulated the levels of PI3K, p-AKT, and p-mTOR. In addition, overexpression of let-7b can further increase the expression level of these proteins compared with A*β*1-40 group. Furthermore, it was observed that the expression of PI3K, p-AKT, and p-mTOR significantly decreased, while autophagy increased and apoptosis decreased after PI3K inhibition. The above results indicated that let-7b overexpression inhibited autophagy and promoted apoptosis via promoting the PI3K/AKT/mTOR signaling pathway, indicating that the PI3K/AKT/mTOR pathway was involved in the imbalance between autophagy and apoptosis.

The article "Inhibiting Autophagy Pathway of PI3K/AKT/mTOR Promotes Apoptosis in SK-N-SH Cell Model of Alzheimer's Disease" was retracted in 2023. Reason: concerns about the peer review.

Beclin-1 is a well-known autophagy inducer that regulates the initiation of autophagosome formation, and its activation can upregulate autophagy. In beclin-1 knockout mice, a significant decrease in expression of beclin-1 leads to reduced neuronal autophagy and ultimately neurodegeneration [33]. In accordance with this, a downregulation of beclin-1 can also be observed in the brains of Alzheimer's patients, especially in the brain regions most susceptible to the pathology of Alzheimer's disease [33]. LC3 is considered as a specific marker of autophagy, while LC3I and LC3II are two key subtypes of LC3. The transformation from LC3I to LC3II indicates autophagy activation [34]. Our research showed that A*β*1-40 treatment inhibited autophagy by inhibiting the transformation from LC3I to LC3II and reducing the level of beclin-1; this effect can be enhanced by let-7b overexpression. Moreover, the effect of let-7b overexpression can be further enhanced by the agonist of PI3K and inhibited by the inhibitor of PI3K, indicating that too low an autophagy level will lead to apoptosis.

Autophagy and apoptosis are two different processes. Autophagy at the basic level can create a cell environment conducive to survival and counteract apoptosis, while abnormal autophagy can promote apoptosis. At present, the mechanism of the autophagy pathway mediating and inhibiting apoptosis is still under investigation. But it is known that autophagy can weaken apoptosis by clearing damaged fragments or degenerated subcellular components. It can maintain genome integrity when cells suffer from metabolic stress, drug toxicity, or radiation damage [35, 36]. Autophagy deficiency can lead to DNA damage, gene amplification, and chromosomal abnormality after metabolic stress in tumor cells [35]. The synergistic effect of autologous defect and altered apoptosis activity may promote malignant differentiation of tumor, resulting in more aggressive cancer cell phenotype and poor prognosis of HCC [37]. Also, autophagy can catabolize organelles and macromolecules, provide nutrition and energy sources for hungry cells, and maintain cell energy balance and cell function. Activation of autophagy in astrocytes deprived of oxygen and glucose is an adaptive mechanism that allows cells to survive longer by delaying the initiation of apoptosis and necrosis [38]. Autophagy limits endoplasmic reticulum (ER) stress by degrading unfolded protein aggregates, and the disorder of ER structure and function would cause ER stress and lead to the accumulation of misfolded proteins. Meanwhile, autophagy can recover protein aggregates and misfolded proteins to maintain ER function, thereby inhibiting ER stress response and subsequent apoptosis [39,40]. What is more, autophagy can promote cell growth and proliferation. It is reported that inhibition of autophagy in human pancreatic cancer cells, leukemia cells, and malignant glioma cells can enhance the death response of these cells to anti-cancer therapies [41]. Inhibition of autophagy increases the anti-tumor effect of histone deacetylase inhibitors in drug-resistant primary chronic myelogenous leukemia and its antiangiogenesis effect in endothelial cells, leading to apoptosis [42, 43]. Regarding the specific signal transduction mechanism, Gentle et al. proposed that autophagy induces apoptosis by modulating the level of interferon-*β* (TRIF) induced by TIR domain of Toll-like receptor (TLR) family [44]. In the rat model of cerebral ischemia, the classical protein kinase C gamma (cPKC*γ*) alleviated the damage of stroke, possibly by downregulating ubiquitin C-terminal hydrolase L1 (UCHL1), upregulating ERK-mTOR pathway, alleviating autophagy and apoptosis, and finally playing a protective role in the brain injury [45]. In the treatment of liver cancer, activation of autophagy through the JNK/beclin-1 pathway can induce apoptosis of cancer cells to achieve partial efficacy [46]. In Parkinson's disease, Piperlongumine (PLG) inhibits apoptosis and induces autophagy by enhancing the phosphorylation of B cell leukemia/lymphoma 2 (BCL 2), which improves neuronal cell activity and mitochondrial function and ultimately improves motor function in Parkinson's mice [47].

The article "Inhibiting Autophagy Pathway of PI3K/AKT/mTOR Promotes Apoptosis in SK-N-SH Cell Model of Alzheimer's Disease" was retracted in 2023. Reason: concerns about the peer review.

## 5. Conclusion

Based on the current research of autophagy and let-7 miRNA in Alzheimer's disease, human neuroblastoma SK-N-SH cell line treated with A*β*1-40 was used in this study to establish an *in vitro* of Alzheimer's disease. In general, autophagy antagonizes apoptosis and promotes cell survival through a series of reactions to damaged organelles. All these indicate that autophagy and apoptosis could interact with each other, and their balance is very important in the course of life.

In a word, this study suggests that A*β*1-40 can induce apoptosis of SK-N-SH cells. In addition, let-7b overexpression can increase the apoptosis of A*β*1-40 treated cells by damaging autophagy, in which process the PI3K/AKT/mTOR signaling pathway is involved. The current results show that let-7b can be used as a promising target and tool for Alzheimer's disease treatment research, but the specific interaction target needs to be further studied. In addition, more samples are needed to ensure the reliability of the experimental results.

## Figures and Tables

**Figure 1:** Relative expression levels of microRNAs in cerebrospinal fluid of patients with Alzheimer's disease.

**Figure 2:** Expression of let-7b in SK-N-SH cells and its influence on cell viability. (a) Expression of let-7b in each group. (b) Cell viability in each group. *n* = 6 per group.  ^*∗*^ ^*∗*^*p* < 0.01 and  ^*∗*^ ^*∗*^ ^*∗*^*p* < 0.001 versus control group; ^##^*p* < 0.01 and ^###^*p* < 0.001 versus A*β*1-40 group, and *p* < 0.01 versus A*β*1-40 + let-7b mimic group.

**Figure 3:** Effect of let-7b on autophagy and apoptosis of SK-N-SH cells treated with A*β*1-40s. (a) Typical Western blot diagram of the expression of each molecule. (b) Statistical graphs of beclin-1 expression in each group. (c) Statistical graphs of LC3II/LC3I expression in each group. (d) Statistical graphs of cleavage caspase 3 expression in each group. (e) Statistical graphs of PI3K expression in each group. (f) Statistical graphs of p-AKT expression in each group. (g) Statistical graphs of p-MTOR expression in each group. *n* = 6,  ^*∗*^ ^*∗*^*p* < 0.01, and  ^*∗*^ ^*∗*^ ^*∗*^*p* < 0.001 versus control group; ^###^*p* < 0.001 versus A*β*1-40 group, and *p*< 0.01 versus A*β*1-40 + let-7b mimic group.

The article "Inhibiting Autophagy Pathway of PI3K/AKT/mTOR Promotes Apoptosis in SK-N-SH Cell Model of Alzheimer's Disease" was retracted in 2023. Reason: concerns about the peer review.

**Figure 4:** Effect of let-7b inhibitor on PI3K/AKT/mTOR signaling pathway. (a) Typical Western blot diagram of the expression of each molecule. (b) Statistical graphs of beclin-1 expression in each group. (c) Statistical graphs of LC3II/LC3I expression in each group. (d) Statistical graphs of cleavage caspase 3 expression in each group. (e) Statistical graphs of PI3K expression in each group. (f) Statistical graphs of p-AKT expression in each group. (g) Statistical graphs of p-MTOR expression in each group. *n* = 6,  ^*∗*^ ^*∗*^*p* < 0.01, and  ^*∗*^ ^*∗*^ ^*∗*^*p* < 0.001 versus control group; ^###^*p* < 0.001 versus A*β*1-40 group, and *p* < 0.01 versus A*β*1-40 + let-7b mimic group.

**Figure 5:** Effect of let-7b agonist on PI3K/AKT/mTOR signaling pathway. (a) Typical Western blot diagram of the expression of each molecule. (b) Statistical graphs of beclin-1 expression in each group. (c) Statistical graphs of LC3II/LC3I expression in each group. (d) Statistical graphs of cleavage caspase 3 expression in each group. (e) Statistical graphs of PI3K expression in each group. (f) Statistical graphs of p-AKT expression in each group. (g) Statistical graphs of p-MTOR expression in each group. *n* = 6,  ^*∗*^ ^*∗*^*p* < 0.01, and  ^*∗*^ ^*∗*^ ^*∗*^*p* < 0.001 versus control group; ^###^*p* < 0.001 versus A*β*1-40 group, and *p* < 0.01 versus A*β*1-40 + let-7b mimic group.

**Table 1:** qPCR primer sequences.

Primer	Sequences
let-7a	5′-UGAGGUAGUAGGUUGUAUAGUU-3′
let-7b	5′-UGAGGUAGUAGGUUGUGUGGUU-3′
let-7c	5′ UGAGGUAGUAGGUUGUAUGGUU-3′
let-7d	5′-AGAGGUAGUAGGUUGCAUAGUU-3′
let-7e	5′-UGAGGUAGGA GGUUGUAUAGUU-3′
let-7f	5′-UGAGGUAGUAGAUUGUAUAGUU-3′
let-7g	5′-UGAGGUAGUAGUUUGUACAGUU-3′
let-7i	5′-UGAGGUAGUAGUUUGUGCUGUU-3′

## Data Availability

The datasets used and/or analyzed during the current study are available from the corresponding author on reasonable request.
